# Diabetic Nephropathy: Challenges in Pathogenesis, Diagnosis, and Treatment

**DOI:** 10.1155/2021/1497449

**Published:** 2021-07-08

**Authors:** Nur Samsu

**Affiliations:** Division of Nephrology and Hypertension, Department of Internal Medicine, Medical Faculty of Universitas Brawijaya-Saiful Anwar General Hospital, Malang, Indonesia

## Abstract

Diabetic nephropathy (DN) is the leading cause of end-stage renal disease worldwide. Chronic hyperglycemia and high blood pressure are the main risk factors for the development of DN. In general, screening for microalbuminuria should be performed annually, starting 5 years after diagnosis in type 1 diabetes and at diagnosis and annually thereafter in type 2 diabetes. Standard therapy is blood glucose and blood pressure control using the renin-angiotensin system blockade, targeting A1c < 7%, and <130/80 mmHg. Regression of albuminuria remains an important therapeutic goal. However, there are problems in diagnosis and treatment of nonproteinuric DN (NP-DN), which does not follow the classic pattern of DN. In fact, the prevalence of DN continues to increase, and additional therapy is needed to prevent or ameliorate the condition. In addition to conventional therapies, vitamin D receptor activators, incretin-related drugs, and therapies that target inflammation may also be promising for the prevention of DN progression. This review focuses on the role of inflammation and oxidative stress in the pathogenesis of DN, approaches to diagnosis in classic and NP-DN, and current and emerging therapeutic interventions.

## 1. Introduction

Diabetic nephropathy (DN) is one of the most frequent and severe complications of diabetes mellitus (DM) and is associated with increased morbidity and mortality in diabetic patients [1]. In the US, the number of diabetic patients starting treatment for end-stage renal disease (ESRD) significantly increased from more than 40,000 in 2000 to more than 50,000 in 2014 [2]. In China, the incidence and prevalence of DN have also increased dramatically over the past decade. The estimated number of diabetic patients with chronic kidney disease (CKD) in China reaches 24.3 million [3]. Overall, the prevalence of diabetes globally is growing rapidly, especially in developing countries [4]. With the increasing prevalence of diabetes, the prevalence of DN is also predicted to increase, if there is no immediate improvement in the clinical strategy of prevention of DN [5, 6].

DN develops after latency periods that may vary by several years in approximately one-third of patients with diabetes. It is still a matter of controversy whether individuals should be screened to find microalbuminuria or screened to predict DN, known as the personalized medicine approach, so as to allocate resources with more intensive therapy and early preventive measures only to the individuals most at risk [7]. At the time of microalbuminuria, there has been advanced glomerulopathy [8, 9]; on the other hand, a large number of patients with microalbuminuria can regress to normoalbuminuria [10]. Diagnosing DN also faces challenges associated with a number of patients with DN who do not follow the classic pattern of DN [11], as well as the problem of diagnosing DN without retinopathy [12], whose prevalence reaches 40% [13]. Nonproteinuric DN and DN without retinopathy are more common in type 2 DM patients. Because renin-angiotensin system (RAS) blockade therapy is usually initiated only after persistent albuminuria [7], the absence of albuminuria can make it difficult to determine the right time to initiate intensive therapeutic interventions.

The pathogenesis of DN is very complex and is still not fully understood, resulting in poor therapeutic outcomes. Standard therapy, with strict blood sugar and blood pressure control, has been shown to be unable to stop DN progression to ESRD [14] and DN-related mortality [15]. Improving understanding and exploring the pathogenic mechanisms of DN is important in developing new strategies for treating DN. There are many pathways and mediators involved in the development and progression of DN [16], including oxidative stress, angiotensin II (Ang-II), and inflammatory processes, which are recently considered to play an important role [17]. Understanding the key features of the inflammatory mechanisms involved in the development and progression of DN also allows identification of new potential targets and facilitates the design of innovative anti-inflammatory therapeutic strategies [17]. This review discusses the pathogenesis of DN, in particular, the role of oxidative stress, Ang-II, and inflammation as well as current and potential future therapeutic developments including those targeted on inflammation.

## 2. Pathogenesis of Classic Diabetic Nephropathy

The pathogenesis of DN development and progression is complex and multifactorial with the involvement of many pathways and mediators [18]. Conventionally, the developmental mechanism of DN is the result of abnormal homeostasis, which includes hemodynamic abnormalities, metabolic disorders, and hormone synthesis such as Ang-II [16]. Renin-angiotensin-aldosterone system (RAAS), advanced glycation end product (AGE) formation, activation of transforming growth factor-*β*1 (TGF-*β*1), connective tissue growth factor (CTGF), protein kinase C (PKC), mitogen-activated protein kinase (MAPKs), and reactive oxygen species (ROS) are important pathways to the development and progression of DN. Each pathway causes damage via multiple mediators or interacts with other pathways. There is a great deal of overlap between pathways and mediators; for example, Ang-II causes injury through oxidative stress, and conversely, oxidative stress causes injury through RAAS. Nicotinamide adenine phosphate dehydrogenase (NADPH) oxidase increases TGF-*β*, and conversely, TGF-*β* increases ROS through activation of NADPH oxidase. This is why the exact pathogenic mechanism and molecular incidence of DN are still not fully understood and the contribution of each pathway in inducing DN is not certain [15].

### 2.1. Role of Oxidative Stress

The role of oxidative stress in DN has been noted by the observation that inhibition of oxidative stress improves a feature associated with streptozotocin-induced DN [19]. Conventionally, oxidative stress is a condition of oxidative damage to tissues due to an imbalance between oxidants and antioxidants [20]. Oxidative stress is a common product of many pathways that are involved in the pathogenesis of DN [15], including hyperglycemia itself. Increased ROS due to hyperglycemia is central to the pathogenesis of DN. In diabetes, the main sources of ROS include the polyol chain, AGE, and NADPH oxidase (Nox) [21]. Isoform Nox 4 is an enzyme that plays the most important role in the production of ROS in the kidneys [22]. Besides, through NADPH oxidase, ROS is also produced through lipoxygenase, uncoupled nitric oxide synthase, xanthine oxidase, and mitochondrial respiratory chain dysfunction [20]. Hyperglycemic-induced oxidative stress is believed to increase levels of proinflammatory proteins by infiltrating macrophages that secrete inflammatory cytokines that cause local and systemic inflammation [23].

The mechanisms of damage induced by oxidative stress can occur directly or indirectly. Oxidative stress can cause direct damage to podocytes, mesangial cells, and endothelial cells, resulting in proteinuria and tubulointerstitial fibrosis [24, 25] This can occur because the glomerulus is a part of the nephron that is more sensitive to oxidative injury than the other parts of the nephron [21]. Hyperglycemia is known to be responsible for deoxyribonucleic acid (DNA), lipid, and protein damage, and the degree of damage has been associated with hyperglycemic-induced ROS production rates and consequently oxidative stress [26]. Meanwhile, indirectly, oxidative stress can activate other pathogenic pathways to cause injury; on the other hand, other pathogenic pathways can cause injury through oxidative stress [27]. Oxidative stress is also associated with metabolic and hemodynamic changes in the kidney, both of which have adverse synergistic effects [28]. Oxidative stress induced by chronic hyperglycemia can induce increased Ang-II levels, PKC activation, and TGF-*β* expression, which, in turn, have also been implicated as important prooxidative stress stimulants [22, 29]. An increase in oxidative stress together with an increase in Ang-II levels will activate TGF-*β*, which in turn stimulates the synthesis of the mesangial matrix. Increased Ang-II will increase renal ROS production through activation of NADPH oxidase. TGF-*β* is also involved in the production of ROS mediated by NADPH oxidase in mesangial cells that are exposed to high glucose levels. The continuous increase and activation of TGF-*β* due to increased production of ROS cause excessive remodeling of the extracellular matrix in the mesangium and promotes fibrotic processes in the tubular interstitium [21].

### 2.2. Role of Renin-Angiotensin-Aldosterone System

The renin-angiotensin-aldosterone system plays (RAAS) an important role in the progression of renal disease, and it has been shown that inhibition of RAAS can inhibit the progression of CKD which is characterized by decreased proteinuria and well-maintained renal function [30]. In diabetes, the role of RAAS has been widely studied in relation to changes in intraglomerular hemodynamics as well as structural changes in both the glomerulus and tubulointerstitium [31, 32]. Podocyte cells have been shown to produce many components of RAAS and express RAAS receptors, including Ang-II receptors (AIIR), mineralocorticoids, and prorenin. It is an important function of podocytes, shown to be regulated by Ang-II type 1 receptors (AT1R) [30].

#### 2.2.1. Role of Angiotensin II

Based on existing evidence, it shows that Ang-II is a cytokine that has many effects on the kidneys [33], through systemic effects and local activation of the RAS in the kidneys [32]. This suggests that Ang-II functions beyond its classical function as a hemodynamic mediator. In addition, there is increasing evidence that oxidative stress, inflammation, and fibrosis are the main links in the development and progression of disease. Oxidative stress is the initial part of DN and activates various pathological pathways in almost all cell types in the kidney (endothelial, mesangial, epithelial, tubular cells, and podocytes) [33]. In general, it can be concluded that Ang-II is a “master” molecule which has a central role in kidney injury, whereas oxidative stress is an integral part of cell damage. Nonetheless, several studies with therapeutic approaches targeted at oxidative stress and Ang-II have uncertain results [34–38].

#### 2.2.2. Role of Renin-Angiotensin System Local Intrarenal

In addition to circulating renin-angiotensin, many tissues such as the uterus, placenta, blood vessels, heart, brain, and, especially the adrenal cortex and kidneys, have local RAS [31]. Renal cells are able to synthesize renin, renin receptors, angiotensin receptors [39], and Ang-II locally independent of systemic RAS [40], so that the kidneys are able to maintain high intrarenal levels of Ang-II. Even the interstitial renal Ang-II levels are 1000-fold higher than in the plasma [41], so that intrarenal RAS is believed to play the major damaging role. In fact, high glucose is known to stimulate renin and Ang-II synthesis in mesangial cells (MCs) [42, 43]. Intrarenal Ang-II has several effects that can contribute to the development of kidney injury, such as increased glomerular capillary pressure and permeability (causing proteinuria), stimulation of renal cell proliferation and hypertrophy, synthesis of cytokines and extracellular matrix (ECM), and promotion of macrophage infiltration and inflammation [44, 45]. Evidence from studies has shown that Ang-II blockade has benefits beyond its blood pressure-lowering effect. At DN, although systemic renin levels are low, it turns out that the blockade effect on RAS can slow disease progression [32, 46].

### 2.3. Role of Inflammation

It has been shown that immune and inflammatory responses play an important role in the pathogenesis of DN [16], but traditionally, DN has not been considered an inflammatory disease. However, recent evidence shows that inflammation of the kidney is very important in initiating the development and progression of DN. Various reports support the role of interleukin- (IL-) 1, IL-6, and IL-18 in the development of DN [47–49]. Leukocytes, monocytes, and macrophages have been implicated in the pathogenesis of DN, and inflammatory biomarkers have been associated with a risk of developing DN [50].

Persistent inflammation of the circulatory system and renal tissue is an important pathophysiological basis in the development of DN. Inflammation may be activated by metabolic, biochemical, and hemodynamic disorders known to be present in DN [51]. Inflammatory factors, such as IL-6, tumor necrosis factor (TNF-*α*), TGF-*β*1, and IL-18 are elevated in blood [52] and have been shown to be involved in the development and progression of DN [53]. Other studies have shown that the levels of this substance increase with the development of nephropathy and are independently associated with urinary albumin excretion [47]. The degree of accumulation of inflammatory cells in the kidney is closely related to DN [54]. On the other hand, in experimental DN, inhibition of the mobilization of inflammatory cells into the kidney has been shown to have a protective effect [55]. This condition suggests that inflammation may be an important pathogenic factor in the development and progression of DN. Proinflammatory and fibrogenic cytokines that are synthesized and secreted by these cells in the local microenvironment can directly damage the renal architecture and then trigger the epithelial-to-mesenchymal transition (EMT) process [56], which in turn results in ECM accumulation. In addition to the synthesis of proinflammatory cytokines, in diabetic animals and kidney cells of diabetic patients, the expression of chemoattractant cytokines and adhesion molecules is also upregulated. These molecules are key mediators of kidney injury due to their ability to attract circulating leukocytes and facilitate the transfer of these cells into kidney tissue. These infiltrated cells are also a source of cytokines and other mediators that contribute to the development and progression of kidney injury, as well as to strengthen and perpetuate inflammatory reactions that have occurred [16].

#### 2.3.1. Role of Transcription Factors and Protein Kinase on Inflammation

*(1) Role of NF-κB*. One of the key elements involved in the inflammatory process in DN is nuclear factor-*κ*B (NF-*κ*B), which is a ubiquitous transcription factor that is activated by many DN inflammatory mediators, such as AGEs, hyperglycemia, and mechanical stress. Furthermore, NF-*κ*B regulates inflammatory cytokines, chemokines, and cell adhesion proteins, which contribute to kidney injury in DN [57]. One of the reasons NF-*κ*B is an important “first respondent” to DN is that it is constantly present in cells even when in an inactive state. Hence, the activation of the pathways involved does not require protein synthesis from these transcription factors, thus enabling them to activate more rapidly. One of the main pathways that respond to and transduce inflammatory signals is the *Janus kinase*/signal transducers and activators of transcription (JAK-STAT) pathway. JAK-STAT is a signaling pathway associated with intracellular cytokines that serve as the main mediator between paracrine stimulation and nuclear receptors. Cytokines and hyperglycemic conditions can activate important mechanisms regulating cell activation, proliferation, recruitment, migration, and differentiation [18]. There is increasing evidence that JAK-STAT plays a central role in the pathogenesis of DN. Early DN patients have reported upregulation of JAK-STAT in glomerular cells. Likewise, tubulointerstitial expression of various JAK and STAT isoforms increases with disease progression and is inversely correlated with estimated-glomerular filtration rate (eGFR). NF-*κ*B, which is a key transcription factor in the inflammatory process in DN, is activated via JAK-STAT. In resident kidney cells, NF-*κ*B is activated rapidly by a variety of stimuli, including hyperglycemia, AGE, mechanical stress, ROS, inflammatory cytokines, Ang-II, and albuminuria. After being activated, NF-*κ*B will stimulate transcription of proinflammatory cytokines, chemokines, and adhesion molecules [57].

*(2) Role of Nrf2*. The transcription factor erythroid nuclear factor 2-related factor 2 (Nrf2) is one of the most important regulators of oxidative stress. Nrf2 regulates the expression of antioxidant cytoprotective genes that attenuate systemic oxidative excess [16]. Under normal physiological conditions, Nrf2 is constitutively ubiquitinated and degraded by proteasomes through interaction with its inhibitor, namely, Kelch-like ECH-associated protein 1 (Keap1). Oxidative stress or electrophilic compounds stabilize Nrf2 by counteracting Keap1 interactions with Nrf2, which causes rapid translocation of Nrf2 into the nucleus to then bind to antioxidant-responsive elements (ARE). This in turn leads to increased transcription of genes coding for antioxidants and detoxifying enzymes such as NAD(P)H : quinine oxidoreductase 1 (NQO1), heme oxygenase-1 (HO-1), *γ*-glutamyl cysteine synthetase (*γ*-GCS), and GST. One of the most attractive features of targeting the Nrf2/Keap1 pathway is that Nrf2 activation leads to upregulation of a wide variety of antioxidant enzymes, rather than relying solely on a single antioxidant enzyme [58]. The Nrf2-/- mice suffered significantly more severe kidney injury than the wild-type mice, and this evidence supports a protective role for Nrf2 in kidney disease [59].

*(3) Role of Protein Kinase*. PKC isoform activation is involved in the pathogenesis of DN. This has been proven by Menne et al. in 2004 in PKC-*α*-/- experimental animals with hyperglycemia conditions [60]. There was almost no albuminuria in mice with PKC-*α*-/- diabetes, as well as decreased VEGF and receptor expression, while TGF-*β* was not affected. These findings indicate that glomerular hypertrophy and albuminuria are regulated by a different mechanism. Albuminuria is mediated by PKC-*α* through downregulation of proteoglycan on MBG and regulation of VEGF expression [61]. The role of PKC-*β* isoform on DN pathogenesis was investigated by Ohshiro et al. in 2006 using mice without PKC-*β* (PKC-*β*-null mice) [62]. PKC-*β* activation can induce renal dysfunction through increased expression of p47phox, Nox-2, Nox-4, endothelin-1, VEGF, TGF-*β*, CTGF, and oxidant production [60].

PKC-*α* activation was associated with the occurrence of albuminuria in DN, but with PKC-*α* inhibition, renal and glomerular hypertrophy persisted. This can occur because the expression of TGF-*β* is not reduced [61]. In contrast, PKC-*β* plays an important role in DN through tubular hypertrophy, mesangial expansion, and glomerular enlargement by reducing TGF-*β*, CTGF, and matrix molecular expression, but it does not prevent albuminuria [60]. A randomized, double-blind, placebo-controlled study assessing the effect of ruboxistaurin, a selective PKC-*β* inhibitor, for 1 year in type 2 diabetic patients with nephropathy found a renoprotective effect through reducing albuminuria and maintaining GFR for more than 1 year [62]. Activation of PKC-*α* and PKC-*β* isoforms is associated with increased NADPH activity and production of NADPH-dependent superoxide, which represent a common pathway among these PKC isoforms in inducing kidney damage [60, 63]. Overall, the mechanisms by which these PKC isoforms induce the progression of DN are very complex [64]. It seems that the selective selection of inhibition of complement control protein (CCP) isoforms plays an important role in DN management.

#### 2.3.2. Relationship between Inflammation and Oxidative Stress

Several studies have supported an interdependent relationship between inflammation and oxidative stress [65, 66]. Inflammation and oxidative stress are closely related to interdependent pathophysiological processes. The interdependence of inflammation and oxidative stress is simply illustrated with great interest by Biswas (Figure 1) [67]. However, in reality there are many other redox-sensitive signal transduction pathways such as c-Jun N-terminal kinase (JNK) and p38 MAP kinase and transcription factor activator protein 1 (AP-1) which also participate to set up a vicious cycle between inflammation and oxidative stress [68]. If oxidative stress appears as a major abnormality in an organ, inflammation will eventually develop and will further accentuate the oxidative stress. Conversely, if inflammation is the main event, oxidative stress will develop as a consequence which will further exaggerate the inflammation [68]. Therefore, the identification of the primary disorder can be of great clinical importance, since treatment of the primary disorder will most likely ensure continued relief from the problem. Nonetheless, identification of the primary disorder is not easy because oxidative stress and inflammation are closely related and are interdependent pathophysiological events [67].

Relatively, the same thing happens in DN; it is difficult to determine the primary abnormality. What is clear is that DN has an increase in serum IL-6 and IL-18 levels [69, 70], and this serum IL-6 level is parallel with the severity of albuminuria [69] and also correlates with morphological changes in DN, such as thickening of glomerular basement membrane (GBM) [71]. IL-18 can induce the release of interferon-*γ* (IFN-*γ*) and the production of other inflammatory cytokines, such as IL-1 and TNF-*α* [72]. In diabetic patients with microalbuminuria or albuminuria, the IL-6 and IL-18 levels were increased compared to patients without albuminuria [70]. Other studies have also shown that IL-18 levels in urine and serum as well as serum IL-6 levels are also significantly increased in type 2 diabetes patients compared to controls. Albuminuria was independently positively correlated with serum and urine IL-18 levels [73]. In the DN model, there was an increase in TNF-*α* expression in the epithelial cells of the proximal tubule and glomerulus [74]. Through NF-*κ*B signaling, TNF-*α* can induce cytokine transcription that affects cell survival, proliferation, adhesions, inflammatory responses, and apoptosis [75]. In addition, as a pleiotropic cytokine, TNF-*α* contributes to DN development through several mechanisms, including decreased GFR, vasoconstriction due to increased endothelin-1 (ET-1) production, and impaired glomerular filtration barrier and proteinuria. Increased TNF-*α* production can also result in oxidative stress, via NADPH activation, in mesangial cells. TNF-*α* is also thought to play a role in apoptosis and direct cytotoxic effects on glomerular cells [57].

Based on the description above, it has been proven that the inflammatory process plays an important role in the pathogenesis of DN. Inflammation in DN is probably activated by metabolic, biochemical, and hemodynamic disturbances that are known to be present in DN [51]. On the other hand, as in the previous explanation, the increase in ROS due to hyperglycemia is central to the pathogenesis of DN [22, 29], and ROS plays an important role in the induction and progression of DN [29, 76]. It is clear that oxidative stress and inflammation, as well as their interactions, have important roles in the pathogenesis and development of CKD [77]. Both increase kidney injury through damage to molecular components [78]. The main pathological mechanisms linking oxidative stress, inflammation, and progression of CKD include early kidney injury by intra- and extracellular oxygen-derived radicals and the resulting inflammation [78]. The kidney is the target organ as well as the organ that is involved in increasing AGE [79, 80]. The occurrence of inflammation in DN can also occur through NF-*κ*B activation induced by an increase in AGE, which will then be followed by an increase in ROS production [81]. Excessive production of ROS corresponds to activation of NF-*κ*B and inflammatory cytokines, which are important in the pathogenesis of DN [82].

## 3. Approaches to Diagnosis of Classic Diabetic Nephropathy

### 3.1. Screening for Diabetic Nephropathy

Conventionally, the natural history of DN consists of 5 stages, mainly based on the proposal by Mogensen et al. [83], with microalbuminuria being the first disorder to occur in individuals suffering from this complication. This is followed by macroalbuminuria and decreased kidney function. On this basis, screening and diagnosis of DN is still based on the albuminuria assessment.

Based on the (ADA) recommendations, screening is carried out for everyone with type 2 diabetes by measuring renal function and albuminuria at diagnosis and annually thereafter; whereas in type 1 DM, it starts after 5 years of diagnosis. However, because the prevalence of microalbuminuria before 5 years in type 1 DM can reach 18% [84], it is advisable to do screening since 1 year of diagnosis. In patients with type 2 diabetes, 7% of patients had microalbuminuria when diagnosed with diabetes [85]. If the screening test does not reveal microalbuminuria, then the screening should be repeated annually for both type 1 and type 2 diabetes patients [86]. Albuminuria can be measured using spot urine measuring albumin-creatinine ratio (ACR) or 24-hour urine, while renal function is recommended using a serum creatinine basis using (CKD-EPI) [87]. If an increase in albuminuria is detected, this should be confirmed on repeat testing over 3 to 6 months; a minimum of two elevated ACR levels more than 3 months apart are required before an individual is considered to have increased albuminuria [88]. Patients with micro- and macroalbuminuria should undergo an evaluation regarding the presence of comorbid associations, especially retinopathy and macrovascular disease.

### 3.2. Diagnosis of Classic Diabetic Nephropathy

The definition of DN is based on current guidelines using four main criteria: a decline in renal function, diabetic retinopathy, proteinuria, and a reduction in GFR [89]. However, the hallmark of established DN is persistent albuminuria, with coexisting retinopathy and no evidence of alternative kidney disease [87]. Practically, DN is a clinical syndrome in DM patients characterized by persistent albuminuria (>300 mg/day or >200 *μ*g/min) at 2 out of 3 examinations within 3-6 months, a progressive decrease in GFR, and hypertension [90].

Basically, natural development of DN differs based on the type of diabetes and the presence of albuminuria (30-300 mg/day). In type 1 diabetes mellitus, DN rarely manifests within the first 10 years after diagnosis, but between 10 and 20 years, the incidence of DN is approximately 3% per year [91]. After 20 years, the incidence rate declines so that people with normal renal function and normal urinary albumin excretion after 30 years of type 1 diabetes mellitus (T1DM) are at lower risk of developing DN [92]. Therefore, the risk of developing DN varies between individuals and is not only dependent on duration of T1DM but is also influenced by other factors [87].

## 4. Diabetic Nephropathy Nonproteinuric

Classically, DN is characterized by the appearance of proteinuria followed by a progressive decline in renal function. However, some diabetic patients develop decreased renal function and vascular complications without proteinuria, known as nonproteinuric DN (NP-DN) [15]. Even based on a survey in the general population, most of patients with diabetes and CKD have no albuminuria [93]. Based on the most recent data, it was found that the opposite temporal trend in the prevalence of albuminuria and a decrease in eGFR in diabetic patients, i.e., despite regression of microalbuminuria (decreased prevalence of albuminuria), the decline in GFR continued [94, 95]. This increased divergence between albuminuria and decreased eGFR differs from the classic view, that albuminuria always precedes and leads to a progressive decrease in GFR. This suggests that the initiation and progression of decreased renal function may also occur independently of the development of albuminuria. This concept is supported by the emergence of two new phenotypes, i.e., nonalbuminuric/proteinuric kidney disorders (NP-DN) and progressive renal decline [96]. Albuminuria and decreased eGFR can occur and continue either together or separately as complementary or “twin” manifestations of DN [97]. So, there are two main pathways for the onset and progression of DN, i.e., albuminuric and nonalbuminuric. The prevalence of NP-DN in type 2 DM ranges from 45 to 70%, while based on the latest data, its prevalence in type 1 DM is from 50 to 60% [96].

### 4.1. Pathogenesis of Nonproteinuric Diabetic Nephropathy

In general, NP-DN is caused by abnormalities in the vascular or predominantly tubulointerstitial abnormalities [98, 99], although it can also be a typical disorder [100, 101]. NP-DN pathophysiological investigations should provide additional insight into cardiovascular factors affecting kidney function and disease and provide new treatments for the vascular complications seen in diabetic patients [17]. There are several possibilities for this NP-DN, including the accompanying vascular disease (there is an increase in interlobar artery vascular resistance) [102] which causes damage to glomerular and tubular structures and interstitial fibrosis [103]: the result of previous episodes of acute kidney injury (AKI), which is related to the inherent susceptibility of diabetic patients [104]; the existence of a well-preserved tubule that leads to a significant reabsorption of albumin from the glomerular filtrate, thus resulting in a diminished albumin excretion into normoalbuminuric levels [102]; and an increase in intrarenal arteriosclerosis as opposed to classical glomerulosclerosis changes present in albuminuric subjects [104]. The main contributing factors to progression to ESRD are AKI, as has been proven by Thakar et al. in 2011. In 2019, Sykes et al. found that AKI events were associated with progression to renal replacement rate and also with a greater severity of subsequent AKI [105, 106]. This may explain why some DN patients have an early decline of GFR with a minimal amount of albuminuria.

In addition, there are other factors that also play a role: (1) Increased levels of uric acid, which can damage vascular elements and cause endothelial dysfunction through various mechanisms, including activation of the Toll-like receptor pathway [107, 108]. Uric acid can also induce renal inflammation, proliferation of vascular smooth muscle cells, and activation of the RAS [109–112]. (2) Increased concentration of serum TNF-*α* [113]. TNF-*α* is a major mediator of inflammation and is involved in AKI, regulation of blood pressure, blood flow, inflammation in the renal blood vessels [114–116], and apoptosis [113]. Thus, elevated levels of TNF-*α* can alter renal blood vessels and damage the kidneys. Others that may play a role are increased levels of osteoprotegerin and vascular endothelial growth factor (VEGF), which function in inflammation and angiogenesis, respectively [117].

With regard to prognosis, NP-DN has a better prognosis than DN with significant proteinuria. This is in accordance with the understanding so far, that the degree of proteinuria is a strong predictor of the risk of progression [101]. However, compared with no kidney disease, NP-DN was a significant risk factor for death and major cardiovascular disease [118].

### 4.2. Diagnosis of Nonproteinuric Diabetic Nephropathy

The diagnosis of NP-DN is based on an increase in the Renal Resistive Index (RRI), which measures renal vascular resistance. RRI measurements have been shown to be reliable for detecting and monitoring the development of DN and NP-DN [119–121]. A study in diabetic patients showed an increased RRI value in diabetic patients without proteinuria or renal atherosclerosis [122]. Therefore, ultrasound sonography provides an effective method to screen, identify, and monitor hemodynamic and morphological changes in DN patients [122]. Furthermore, diabetic patients who are identified as being at high risk for developing DN may qualify for pharmacological treatment, which may prevent the onset of DN before the onset of proteinuria [123].

## 5. Risk Factors of Progressivity of Diabetic Nephropathy

Hyperglycemia, hypertension, obesity, smoking, race, men, dyslipidemia, age, and genetic factors are the main risk factors for the development and progression of DN [124–126]. The incidence of DN is higher for African Americans, Asians, and Native Americans than for Caucasians [86]. Siblings of diabetic patients with nephropathy have a 3 times greater risk of suffering from the same disease than siblings of diabetic patients without nephropathy [127]. The development of DN is generally divided into five stages. It is called microalbuminuria, if the albumin excretion rate is persistent between 30 and 300 mg/day (20-200 mg/min). It is called overt nephropathy if the albumin excretion rate is above 300 mg/day. The presence of albuminuria is associated with an increased risk of cardiovascular disease and progressive kidney disease. Since DN occurred, the rate of reduction in GFR and the adverse effects of hypertension began to appear in patients with type 1 and 2 diabetes. There was a linear decrease in GFR of 2-20 mL/min/year with the progression of DN. In the absence of aggressive intervention, DN will develop into ESRD in 6-7 years on average. The rate of decline in renal function after DN varies between patients and is influenced by additional factors, including blood pressure and glycemic control [128]. Faster development can occur at heavier degrees of albuminuria and hypertension [90]. The presence of retinopathy is also a predictor of faster DN progression [13].

## 6. Indications of Renal Biopsy in Diabetic Patients

Currently, renal biopsy for diagnostic purposes is indicated in cases of atypical presentations that suggest the presence of other renal disorders that may benefit from specific treatment [96]. Although the true prevalence of nondiabetic kidney disease in diabetic individuals may be <10% [129], this possibility should always be considered and a kidney biopsy must be performed in the presence of certain clinical criteria: (1) short-duration type 1 diabetes, (2) diagnosis of autoimmune disease, (3) mild or absent retinopathy, (4) red cell casts in urine (active urinary sediment), (5) significant and persistent proteinuria [130, 131], and (6) family history of nondiabetic forms of kidney disease [87].

## 7. Approaches to Management of Diabetic Nephropathy

In classic DN patients, standard therapy still focuses on glucose and blood pressure control, with the target of halting DN progression and regression of albuminuria. This albuminuria regression target is based on the assumption that decreased albuminuria in diabetic individual results in better renal and CVD outcomes [132]. However, this approach has been shown to only be able to slow down the rate of development but not to stop or reverse the disease [14], so that the prevalence of DN is still increasing. Based on a series of cross-sectional studies conducted in a Japanese diabetic population, it has been demonstrated that the prevalence of DN has increased from 18.5% in 1996 to 25.6% in 2014 [95]. However, albuminuria remains a strong predictor of eGFR decline and a main target of renoprotective therapy, especially in the setting of moderate-to-severe impairment of renal function [96]. One of the most important risk factors for the development of kidney disease in diabetic patients is the onset and persistence of proteinuria [132]. In addition to the above approaches, other nonspecific measures must still be implemented, including weight loss, protein restriction, lipid lowering and smoking cessation [133]. Overweight and obesity increase hyperfiltration and specific hormonal dysregulation associated with adipokines that play a role in DN [134]. Weight loss in obese diabetic patients has been shown to reduce albuminuria [135].

In NP-DN patients, the main underlying abnormality is vascular, the principle of targeted therapy as well as cardiovascular risk factors that is seen in diabetic patients. In recent years, pharmacological alternatives for DN, such as heparin or heparin derivatives (Sulodexide) and antibody therapy, have been proposed for treating glomerular vascular syndrome [17].

### 7.1. Blood Glucose Control

#### 7.1.1. Target of Hemoglobin A1c (HbA1c)

Adequate glucose control is a standard foundation in preventing the development and progression of DN. The *United Kingdom* Prospective Diabetes Study (UKPDS) and the *Action in Diabetes and Vascular disease*: *Preterax and Diamicron-MR Controlled Evaluation* (ADVANCE) studies have shown that intensive therapy reduces the risk of diabetic microvascular complications, including DN. The UKPDS study identified a direct association between the risk of diabetes-related complications and glycemic levels, without specifying a “safe” threshold for glycemia [136]. Meanwhile, the ADVANCE study found a nonlinear relationship between HbA1c levels and the risk of microvascular complications. For HbA1c levels < 6.5%, there was no evidence of reduced risk of microvascular complications; whereas, HbA1c > 6.5% was associated with microvascular complications. Each 1% increase in HbA1c was associated with a 40% greater risk of microvascular complications [137]. Based on this research, the recommended target for HbA1c based on ADA is 7.0% [138]. Kidney Disease Outcomes Quality Initiative (KDOQI) recommends individualization in treatment intensity according to patient characteristics to avoid the risk of severe hypoglycemia [139].

#### 7.1.2. Antidiabetic Drug Options

The management of hyperglycemia in CKD, especially those accompanied by a decrease in GFR is a challenge, which requires a more specific understanding, especially in relation to drug choice [96]. DN patients are usually older, with a longer duration of diabetes, more often with comorbidities, so there is a potential for interactions with antihyperglycemic drugs [140]. Drug options are also more limited, although they have increased substantially over the past few decades. Detailed knowledge is required of the choice of drugs that can be used safely and the effect of kidney disease on the metabolism of these drugs. In general, it is recommended to use insulin. However, some oral antidiabetic drugs can still be used with attention adjusted to the patient's GFR. Second generation sulfonylurea groups, such as glipizide and gliclazide, are not contraindicated in patients with renal dysfunction, since they are metabolized by the liver and excreted in the urine as inactive metabolites [141, 142]. More caution is needed when using glipizide if the GFR is <30 cc/minute; be careful of glimepiride at a GFR < 60 cc/minute and avoid it when the GFR is <30 cc/minute, whereas gliclazide can be used without dose adjustment [143, 144]. Repaglinide can be given without dose adjustment (more caution is needed if the GFR is <30 cc/minute) [145]. Incretin-based treatment, dipeptidyl peptidase-4 (DPP-4) inhibitors, and glucagon-like peptide (GLP-1) agonists in general can be used with some drugs requiring dose adjustment, whereas sodium-glucose cotransporter (SGLT2) inhibitors are generally not recommended in patients with GFR < 45 cc/minute [144, 146].

The insulin sensitizers, biguanides and thiazolidinediones, and the inhibitors of *α*-glycosidase are associated with low risk of hypoglycemia [96]. Because metformin is not metabolized by the liver and is excreted unchanged by the kidneys [147], the plasma concentration in patients with renal impairment will increase so that metformin is contraindicated in these individuals. Avoid using metformin at GFR < 30 cc/minute, and it is not recommended as a new therapy for GFR between 30 and 44 cc/minute. Meanwhile, pioglitazone is completely metabolized by the liver, so there is no need to adjust the dose for impaired renal function. Acarbose is metabolized by intestinal bacteria, with the production of several metabolites, and only a small amount of the drug is absorbed. But because the evidence in patients with severe renal insufficiency is still limited, acarbose should be avoided in individuals with very low eGFR [143, 144].

*(1) DPP-4 Inhibitors*. DPP-4 inhibitors are inhibiting the DPP-4 enzyme, increasing levels of endogenous glucagon-like peptide- (GLP-) 1, which promotes insulin secretion but inhibits glucagon secretion, so that blood glucose levels decrease [148]. DPP-4 inhibitors can be used in patients with impaired renal function, although at reduced doses (except for linagliptin, which does not require dose adjustment), they are weight neutral and have a very good safety profile [96]. Recent data suggest that DPP-4 inhibition is associated with a pleiotropic effect on cardiorenal protection. Apart from the glucose-lowering effect, this drug has a renoprotective effect through antioxidant and anti-inflammatory mechanisms, and it is antifibrotic through suppression of TGF-*β*-mediated signaling [149–151]. DPP-4 is expressed in most of the specific organs and cells, with relatively high concentrations and activities found in the kidney, especially in the brush borders of proximal tubular cells [152, 153].

*(2) SGLT2 Inhibitors*. SGLT2 inhibitors are oral hypoglycemic drugs that reduce renal glucose uptake, thereby increasing urinary glucose excretion and reducing hyperglycemia [154]. Based on the EMPA-REG outcome study (Empagliflozin Cardiovascular Outcome Event Trial in Type 2 Diabetes Mellitus Patients), empagliflozin also inhibits the progression of kidney disease, which is characterized by a 39% reduction in worsening nephropathy or cardiovascular death [155]. Renoprotective mechanisms of SGLT2 inhibitors that do not depend on glycemic control include blood pressure control through decreased vascular resistance, weight loss, reduction in intraglomerular pressure so as to prevent the development of glomerular hyperfiltration, and decreased proximal tubular injury biomarkers [156–158]. Hypertension and obesity alone are also risk factors for DN [154]. The CANVAS study (Canagliflozin Cardiovascular Assessment Study) has also shown decreased nephropathy through decreased progression of albuminuria, decreased worsening of GFR, and reduced need for renal replacement therapy or death from kidney causes [159].

### 7.2. Blood Pressure Control

Based on the UKPDS study, a 10 mmHg reduction in systolic blood pressure was associated with a reduction in diabetic microvascular complications, including nephropathy. ADA recommends a blood pressure reduction target of <140/90 mmHg [160], and KDOQI recommends a BP of ≤140/90 mmHg for diabetes without albuminuria, whereas for diabetes with albuminuria it is ≤130/80 mmHg [161]. The 2012 KDIGO guidelines maintain strict blood pressure recommendations for proteinuric patients, regardless of etiology [162]. To control blood pressure, it is recommended to use RAAS inhibitors, i.e., Ang-II receptor blockers (ARBs) or angiotensin converting enzyme (ACE) inhibitors [159]. This recommendation is based on the presence of a lot of research evidence, that inhibition of RAAS is the single most effective therapy to slow the progression of DN to ESRD [159, 163]. Several studies such as IDNT (Irbesartan Diabetic Nephropathy Trial), RENAAL (Reduction in End-Points in Noninsulin-Dependent Diabetes Mellitus with the Ang-II Antagonist Losartan), IRMA-2 (Effect of Irbesartan in the Development of Diabetic Nephropathy in Patients with T2DM), ROADMAP (Randomized Olmesartan and Diabetes Microalbuminuria Prevention), and the Captopril study all demonstrated inhibition of DN progression [163]. However, the combination of ARBs with ACE inhibitors is not recommended, because there is less evidence of a benefit from this combination on cardiovascular disease or DN compared to monotherapy, in addition to the increased incidence of side effects such as hyperkalemia [154]. Based on experimental studies and small-scale clinical studies, nondihydropyridine calcium channel blockers, diltiazem has also been shown to slow the rate of progression of DN, whereas dihydropyridines have varied effects on albumin excretion [163].

## 8. New Potential Therapeutic Strategies

It has been shown that the standard management strategy for DN, which is strict glucose control and blood pressure with RAAS blockade as described above, is only able to slow down the rate of progression but not stop or reverse the disease. Therefore, new drugs targeting DN pathomechanisms, such as oxidative stress and inflammation, have become a major focus for the development of new therapies [164].

### 8.1. Mineralocorticoid Receptor Antagonists

Besides the function of regulating sodium balance through mineralocorticoid receptor activation, aldosterone also has the effect of increasing inflammation and fibrosis [165]. The addition of aldosterone blockers to standard therapy has provided additional benefits in several clinical trials [166, 167]. This drug has shown a slight renoprotective advantage over ACE-inhibitor or ARB therapy [168]. However, the use of mineralocorticoid receptor antagonists (MRA), spironolactone and eplerenone, should be closely monitored as they increase the risk of hyperkalemia, especially in patients with diabetes and CKD.

### 8.2. Endothelin Receptor Antagonists

Endothelin 1 (ET-1) is a strong vasoconstrictor and mitogenic factor that exhibits vasoactive, inflammatory, and profibrogenic properties and has implications for cardiovascular disease and CKD. ET-1 contributes to renal fibrosis through various mechanisms, promotes the accumulation of extracellular matrix components and endothelial cell proliferation, stimulates the epithelial-mesenchymal transition, and increases the production of cytokines and growth factors [169]. In phase III clinical trials, the ET receptor antagonist, avocentan, decreased albuminuria; however, the trial was terminated prematurely due to the drug's effect on significantly increasing fluid overload and the incidence of congestive heart failure. Such side effects may be due to the natriuretic effect of endothelin-B receptor inhibition [170].

### 8.3. Vitamin D Receptor Activators (VDRA)

1,25-Dihydroxyvitamin D3 (1,25(OH)2D3) is a hormonal form of vitamin D, which is an endocrine hormone with various physiological functions [171]. It has been shown that 1,25(OH)2D3 functions as a negative endocrine regulator of RAS [172]. Activation of vitamin D receptors has anti-inflammatory, immunological, and nephroprotective action [173]. On that basis, therapy with VDRA (paricalcitol or calcitriol) may have some protection in DN. Based on findings from the Third National Health and Nutrition Examination Survey (NHANES III) in the population, a decrease in 25(OH)D2 concentrations is associated with an increased prevalence of albuminuria and there is an independent relationship between VD and DN deficiency. With progressive DN, the VD insufficiency becomes more severe [174]. Based on the subanalysis of PRONEDI's research, it shows that lower 25-OH-vitamin D levels have been independently linked to DN progression [175].

A systematic review including clinical trials of the effects of active vitamin D (both paricalcitol and calcitriol) on the control of proteinuria in CKD patients concluded that these drugs provide a significant reduction in proteinuria in addition to blockade of the renin-angiotensin system [176]. An important mechanism underlying the renoprotective effect of VDR activator (VDRA) is related to protection against podocyte injury and inhibition of podocyte apoptosis [177]. This is evidenced by the growing evidence of the last few years which showed that podocytes express VDR, and the VD/VDR signaling pathway has potent renal protective activity against DN [178]. Another study also reported that 1,25(OH)2D3 can reduce hypercorrection levels of fibroblast growth factor 23 (FGF23) which is also a risk factor for DN development and can damage podocytes [179]. Based on the above studies, this strongly supports the recommendation of vitamin D supplementation for the prevention and management of DN.

### 8.4. Therapies Targeting Inflammation

Pentoxifylline (PTF) is a methylxanthine-derived phosphodiesterase inhibitor which is used primarily to treat peripheral vascular disease, as it has beneficial effects on microcirculatory blood flow [18]. A meta-analysis reported a substantial antiproteinuric effect of PTF in patients with DN, whose effect was thought to be due to a decrease in proinflammatory cytokines [180]. A randomized controlled trial reported that adding a low dose of pentoxifylline (400 mg daily) in 50 patients with T2DM who received multiple RAS blockade therapy (losartan and enalapril) resulted in a decrease in urinary protein excretion from 616 mg/day at baseline to 192 mg/days at 6 months (*p* < 0.001) [181]. Whereas in the Pentoxifylline for Renoprotection in Diabetic Nephropathy study (PREDIAN trial) which also evaluated the effect of PTF in type 2 DM patients with CKD stages 3-4 with residual albuminuria despite maximized RAS inhibitor treatment, it shows that after 24 months of therapy, eGFR decreased by 2.1 ± 0.4 mL/minute/1.73 m^2^ in the treatment group, and there was a significant difference (*p* < 0.001) compared to a decrease of 6.5 ± 0.4 mL/minute/1.73 m^2^ in the control group. The difference between groups in the change in albuminuria between groups was also significant (5.7 vs. -14.9%; *p* = 0.001) [182].

High glucose causes a proinflammatory response in tubular cells and podocytes which is characterized by chemokine secretion that triggers renal inflammation [183]. Emapticap Pegol is a monocyte chemoattractant protein*-*1/chemokine (C-C motif) ligand 2 (MCP-1/CC2) antagonist evaluated in a phase 2, placebo-controlled trial in DN patients with residual macroalbuminuria while on RAS inhibitor therapy. After 12 weeks, the urinary albumin-to-creatinine ratio (UACR) was 29% lower compared to baseline, but there was no significant difference with the placebo group. A difference of 26% (*p* = 0.06) between emapticap and placebo was seen 8 weeks after discontinuation of treatment [60]. Whereas CCX140-B is a selective CCR2 inhibitor. In a double-blind, placebo-controlled trial in DN patients with proteinuria, eGFR 25 mL/minute/1.72 m^2^ or higher, and who received RAS inhibitors, CCX140-B therapy was administered at a dose of 5 mg or 10 mg. Treatment with a 5 mg dose resulted in a significant 18% reduction in albuminuria compared with the placebo group. This effect lasted for 52 weeks of study [184].

### 8.5. Therapies Targeting Free Radicals

The human body has antioxidants as a defense mechanism that counterbalances the effects of oxidants. Antioxidants are divided into enzymatic and nonenzymatic antioxidants. The main enzymatic antioxidants are superoxide dismutase (SOD), catalase, glutathione peroxidase (GSH-Px), haem oxygenase-1 (HO-1), and thioredoxin. The main nonenzymatic antioxidants are glutathione (GSH), vitamins (vitamins C and E), and *β*-carotene [185, 186]. They are low molecular weight compounds and are found in plasma, extracellular fluid, intracellular fluid, lipoproteins, and membranes [187]. The principle in radical-based therapy is an intervention that can reduce or control the production of ROS and increase endogenous antioxidant activity and/or exogenous antioxidant therapy. Because hyperglycemia is the primary controller of oxidative stress, tight glycemia control remains the cornerstone of current standard therapeutic approaches. Therapy with RAAS blockers has been shown to have therapeutic potential in the treatment of DN. Telmisartan ARB, in addition to reducing albuminuria [188], also has antioxidant properties by increasing the activity of a superoxide-scavenging enzyme, i.e., SOD, by reducing NOX, an enzyme responsible for superoxide production [189, 190].

#### 8.5.1. Resveratrol

Resveratrol is a natural polyphenol compound that has been reported to have beneficial effects on cardiovascular disease, including kidney disease [191, 192]. Resveratrol is a natural antioxidant, which is known to be a strong scavenger of superoxide, hydroxyl radicals, and peroxynitrite [193]. Apart from scavenging ROS, resveratrol also has many protective effects against age-related disorders, including kidney disease, through activation of Sirtuin 1 (SIRT1). Resveratrol is expected to be a useful complementary therapy for preventing kidney injury [191].

#### 8.5.2. Nrf2 Activators

Activation of Nrf2 reduces renal inflammation by suppressing macrophage inflammatory response by blocking the transcription of proinflammatory cytokines including IL-1 and IL-6 [194]. The transcription factor, Nrf2, is a major regulator of redox homeostasis and cellular detoxification responses. Activation of Nrf2 results in a combined upregulation of several antioxidant enzymes and cytoprotective genes, making it an attractive therapeutic target against diabetic complications. In the future, Nrf2 activation is expected to be an important therapeutic strategy in preventing the development of diabetic complications [58]. Bardoxolone methyl is a synthetic triterpenoid activator of the transcription factor Nrf2 and an inhibitor of NF-*κ*B [195]. The BEAM (52-week bardoxolone methyl treatment: renal function in CKD/type 2 diabetes) shows that bardoxolone methyl was associated with improvement in the estimated GFR in patients with advanced CKD and type 2 diabetes at 24 weeks [196]. The improvement persisted at 52 weeks, suggesting that bardoxolone methyl may have promise for the treatment of CKD. The BEACON study also demonstrated the results of bardoxolone methyl inducing an increase in GFR, but this study was discontinued, for safety reasons related to heart failure due to fluid retention [196, 197]. On the other hand, other Nrf2 activators such as dimethyl fumarate are currently used to treat multiple sclerosis [198], as well as research exploring the safety and tolerability of the bardoxolone methyl formulation RTA 402. Thus, the Nrf2 drive for DN cannot be completely dismissed. The successful and safe use of other indications or the observation of better renal outcomes in multiple sclerosis patients may trigger second-round interest in bardoxolone methyl or other Nrf2 activators for DN [199].

## 9. Conclusions

The development and progression of DN are associated with numerous risk factors. In addition, DN patients are usually older, with longer duration of diabetes, and more often with comorbidities, so the therapeutic regimen of DN is usually multifactorial, which includes tight glycemic control, blood pressure control using RAAS inhibitors, lipid-lowering agents, weight loss, protein restriction, and smoking cessation. Although blood glucose and blood pressure levels are well controlled, and nonspecific measures are also implemented, the progression of DN cannot be stopped. Many diabetic patients develop ESRD, and disproportionate spending on health care becomes a tremendous socioeconomic burden on society. Therefore, there is an urgent need to improve the mechanistic understanding of DN and then develop new and effective therapeutic approaches to delay the development of DN. Also, to assess the success of the therapy, the reliable markers used in the progression of DN and ESRD should be identified. The use of this reliable marker is also important because many patients have DN without albuminuria (NP-DN).

In the future, it appears that vitamin D receptor activators (VDRA) and incretin-related drugs for glycemic control (DDP4 inhibitors and GLP-1 agonists) are promising therapies for stopping the progression of DN. Likewise, new drugs targeting DN pathomechanisms, such as oxidative stress, and inflammation have been a major focus for the development of new therapies.

## Figures and Tables

**Figure 1:** When oxidative stress appears as a primary disorder, inflammation develops as a secondary disorder and further increases oxidative stress. On the other hand, inflammation as a primary disorder can cause oxidative stress as a secondary disorder, which can further increase inflammation [67].

## References

[1] Valencia W. M., Florez H. (2017). How to prevent the microvascular complications of type 2 diabetes beyond glucose control. *BMJ*.

[2] Burrows N. R., Hora I., Geiss L. S., Gregg E. W., Albright A. (2017). Incidence of end-stage renal disease attributed to diabetes among persons with diagnosed diabetes—United States and Puerto Rico, 2000-2014. *MMWR. Morbidity and Mortality Weekly Report*.

[3] Zhang L., Long J., Jiang W. (2016). Trends in chronic kidney disease in China. *New England Journal of Medicine*.

[4] Xue R., Gui D., Zheng L., Zhai R., Wang F., Wang N. (2017). Mechanistic insight and management of diabetic nephropathy: recent progress and future perspective. *Journal of Diabetes Research*.

[5] Gheith O., Farouk N., Nampoory N., Halim M. A., Al-Otaibi T. (2015). Diabetic kidney disease: worldwide difference of prevalence and risk factors. *Journal of Nephropharmacology*.

[6] Stenvinkel P. (2010). Chronic kidney disease: a public health priority and harbinger of premature cardiovascular disease. *Journal of Internal Medicine*.

[7] Susztak K., Böttinger E. P. (2006). Diabetic nephropathy: a frontier for personalized medicine. *Journal of the American Society of Nephrology*.

[8] Fioretto P., Steffes M. W., Mauer M. (1994). Glomerular structure in nonproteinuric IDDM patients with various levels of albuminuria. *Diabetes*.

[9] Caramori M. L., Kim Y., Huang C. (2002). Cellular basis of diabetic nephropathy: 1. study design and renal structural-functional relationships in patients with long-standing Type 1 diabetes. *Diabetes*.

[10] Perkins B. A., Ficociello L. H., Silva K. H., Finkelstein D. M., Warram J. H., Krolewski A. S. (2003). Regression of microalbuminuria in type 1 diabetes. *New England Journal of Medicine*.

[11] Chen Y., Lee K., Ni Z., He J. C. (2020). Diabetic kidney disease: challenges, advances, and opportunities. *Kidney Diseases*.

[12] Kramer H. J., Nguyen Q. D., Curhan G., Hsu C. (2003). Renal insufficiency in the absence of albuminuria and retinopathy among adults with type 2 diabetes mellitus. *JAMA*.

[13] Trevisan R., Vedovato M., Mazzon C. (2002). Concomitance of diabetic retinopathy and proteinuria accelerates the rate of decline of kidney function in type 2 diabetic patients. *Diabetes Care*.

[14] Arora M. K., Singh U. K. (2013). Molecular mechanisms in the pathogenesis of diabetic nephropathy: an update. *Vascular Pharmacology*.

[15] Kopel J., Pena-Hernandez C., Nugent K. (2019). Evolving spectrum of diabetic nephropathy. *World Journal of Diabetes*.

[16] Tavafi M. (2013). Diabetic nephropathy and antioxidants. *Journal of Nephropathology*.

[17] Donate-Correa J., Luis-Rodríguez D., Martín-Núñez E. (2020). Inflammatory targets in diabetic nephropathy. *Journal of Clinical Medicine*.

[18] Pérez-Morales R. E., del Pino M. D., Valdivielso J. M., Ortiz A., Mora-Fernández C., Navarro-González J. F. (2019). Inflammation in diabetic kidney disease. *Nephron.*.

[19] Thallas-Bonke V., Thorpe S. R., Coughlan M. T. (2008). Inhibition of NADPH Oxidase prevents advanced glycation end product-mediated Damage in diabetic nephropathy through a protein kinase C- -Dependent pathway. *Diabetes*.

[20] Kao M. P., Ang D. S., Pall A., Struthers A. D. (2010). Oxidative stress in renal dysfunction: mechanisms, clinical sequelae and therapeutic options. *Journal of Human Hypertension*.

[21] Krishan P., Chakkarwar V. A. (2011). Diabetic nephropathy: aggressive involvement of oxidative stress. *Journal of Pharmaceutical Education & Research*.

[22] Brownlee M. (2005). The pathobiology of diabetic complications: a unifying mechanism. *Diabetes*.

[23] Wellen K. E., Hotamisligil G. S. (2005). Inflammation, stress, and diabetes. *Journal of Clinical Investigation*.

[24] Khazim K., Gorin Y., Cavaglieri R. C., Abboud H. E., Fanti P. (2013). The antioxidant silybin prevents high glucose-induced oxidative stress and podocyte injury in vitro and in vivo. *American Journal of Physiology-Renal Physiology*.

[25] Duni A., Liakopoulos V., Roumeliotis S., Peschos D., Dounousi E. (2019). Oxidative stress in the pathogenesis and evolution of chronic kidney disease: untangling Ariadne’s thread. *International Journal of Molecular Sciences*.

[26] Butkowski E. G., Jelinek H. F. (2017). Hyperglycaemia, oxidative stress and inflammatory markers. *Redox Report*.

[27] Tavafi M. (2013). Complexity of diabetic nephropathy pathogenesis and design of investigations. *Journal of Renal Injury Prevention*.

[28] Ceriello A., Morocutti A., Mercuri F. (2000). Defective intracellular antioxidant enzyme production in type 1 diabetic patients with nephropathy. *Diabetes*.

[29] Forbes J. M., Coughlan M. T., Cooper M. E. (2008). Oxidative stress as a major culprit in kidney disease in diabetes. *Diabetes*.

[30] Wennmann D. O., Hsu H.-H., Pavenstädt H. (2012). The renin-angiotensin-aldosterone system in podocytes. *Seminars in Nephrology*.

[31] Chawla T., Sharma D., Singh A. (2010). Role of the renin angiotensin system in diabetic nephropathy. *World Journal of Diabetes*.

[32] Campbell K., Yacoub R. (2015). Inhibition of RAS in diabetic nephropathy. *International Journal of Nephrology and Renovascular Disease*.

[33] Wada J., Makino H. (2013). Inflammation and the pathogenesis of diabetic nephropathy. *Clinical Science*.

[34] Allam M. M., Nawara H. M., AbdelMaksoud A. A., El-Talees A. E. D. A., Elhamady M. S. (2014). *Nephroprotective Role of Losartan and Vitamin E against Streptozotocin-Induced Diabetic Nephropathy in Rats: Histological and Immunohistochemical Study*.

[35] Alkaaby A. H., Alhelu N. J. A., Almosewi N. A. G. (2017). Nephroprotective effect of vitamin E added to angiotensin receptor blocker in patients with diabetic nephropathy. *Kufa Medical Journal*.

[36] Ma R., Xu Y., Jiang W., Zhang W. (2015). Combination of *Tripterygium wilfordii* Hook F and angiotensin receptor blocker synergistically reduces excretion of urinary podocytes in patients with type 2 diabetic kidney disease. *Biotechnology & Biotechnological Equipment*.

[37] Nie J. M., Li H. F. (2018). Therapeutic effects of *Salvia miltiorrhiza* injection combined with telmisartan in patients with diabetic nephropathy by influencing collagen IV and fibronectin: a case-control study. *Experimental and Therapeutic Medicine*.

[38] Samsu N., Soeharto S., Rifai M., Rudijanto A. (2019). Rosmarinic acid monotherapy is better than the combination of rosmarinic acid and telmisartan in preventing podocyte detachment and inhibiting the progression of diabetic nephropathy in rats. *Biologics: Targets and Therapy*.

[39] Nguyen G., Delarue F., Burcklé C., Bouzhir L., Giller T., Sraer J.-D. (2002). Pivotal role of the renin/prorenin receptor in angiotensin II production and cellular responses to renin. *Journal of Clinical Investigation*.

[40] Lavoie J. L., Sigmund C. D. (2003). Minireview: overview of the renin-angiotensin system—an endocrine and paracrine system. *Endocrinology*.

[41] Nishiyama A., Seth D. M., Navar L. G. (2002). Renal interstitial fluid concentrations of angiotensins I and II in anesthetized rats. *Hypertension*.

[42] Singh R., Singh A. K., Alavi N., Leehey D. J. (2003). Mechanism of increased angiotensin II levels in glomerular mesangial cells cultured in high glucose. *Journal of the American Society of Nephrology*.

[43] Vidotti D. B., Casarini D. E., Cristovam P. C., Leite C. A., Schor N., Boim M. A. (2004). High glucose concentration stimulates intracellular renin activity and angiotensin II generation in rat mesangial cells. *American Journal of Physiology-Renal Physiology*.

[44] Navar L. G., Inscho E. W., Majid S. A., Imig J. D., Harrison-Bernard L. M., Mitchell K. D. (1996). Paracrine regulation of the renal microcirculation. *Physiological Reviews*.

[45] Gilbert R. E., Krum H., Wilkinson-Berka J., Kelly D. J. (2003). The renin-angiotensin system and the long-term complications of diabetes: pathophysiological and therapeutic considerations. *Diabetic Medicine*.

[46] Durvasula R. V., Shankland S. J. (2006). The renin-angiotensin system in glomerular podocytes: mediator of glomerulosclerosis and link to hypertensive nephropathy. *Current Hypertension Reports*.

[47] Navarro J. F., Mora C. (2005). Role of inflammation in diabetic complications. *Nephrology Dialysis Transplantation*.

[48] Suzuki D., Miyazaki M., Naka R. (1995). In situ Hybridization of Interleukin 6 in diabetic nephropathy. *Diabetes*.

[49] Wong C. K., Ho A. W., Tong P. C. (2007). Aberrant activation profile of cytokines and mitogen-activated protein kinases in type 2 diabetic patients with nephropathy. *Clinical & Experimental Immunology*.

[50] Kiritoshi S., Nishikawa T., Sonoda K. (2003). Reactive oxygen species from mitochondria induce cyclooxygenase-2 gene expression in human mesangial cells: potential role in diabetic nephropathy. *Diabetes*.

[51] Lim A. K., Tesch G. H. (2012). Inflammation in diabetic nephropathy. *Mediators of Inflammation*.

[52] Pickup J. C., Chusney G. D., Thomas S. M., Burt D. (2000). Plasma interleukin-6, tumour necrosis factor *α* and blood cytokine production in type 2 diabetes. *Life Sciences*.

[53] Shang J., Wang L., Zhang Y. (2019). Chemerin/ChemR23 axis promotes inflammation of glomerular endothelial cells in diabetic nephropathy. *Journal of Cellular and Molecular Medicine*.

[54] Nguyen D., Ping F., Mu W., Hill P., Atkins R. C., Chadban S. J. (2006). Macrophage accumulation in human progressive diabetic nephropathy. *Nephrology*.

[55] Awad A. S., Kinsey G. R., Khutsishvili K., Gao T., Bolton W. K., Okusa M. D. (2011). Monocyte/macrophage chemokine receptor CCR2 mediates diabetic renal injury. *American Journal of Physiology-Renal Physiology*.

[56] Liu Y. (2011). Cellular and molecular mechanisms of renal fibrosis. *Nature Reviews Nephrology*.

[57] Navarro-González J. F., Mora-Fernández C., Muros de Fuentes M., García-Pérez J. (2011). Inflammatory molecules and pathways in the pathogenesis of diabetic nephropathy. *Nature Reviews Nephrology*.

[58] Tan S. M., de Haan J. B. (2014). Combating oxidative stress in diabetic complications with Nrf2 activators: how much is too much?. *Redox Report*.

[59] Jiang T., Huang Z., Lin Y., Zhang Z., Fang D., Zhang D. D. (2010). The protective role of Nrf2 in streptozotocin-induced diabetic nephropathy. *Diabetes*.

[60] Menne J., Park J. K., Boehne M. (2004). Diminished loss of proteoglycans and lack of albuminuria in protein kinase C-alpha-deficient diabetic mice. *Diabetes.*.

[61] Takebayashi K., Matsumoto S., Aso Y., Inukai T. (2006). Aldosterone blockade attenuates urinary monocyte chemoattractant protein-1 and oxidative stress in patients with type 2 diabetes complicated by diabetic nephropathy. *The Journal of Clinical Endocrinology & Metabolism*.

[62] Ohshiro Y., Ma R. C., Yasuda Y. (2006). Reduction of diabetes-induced oxidative stress, fibrotic cytokine expression, and renal dysfunction in protein kinase Cbeta-null mice. *Diabetes*.

[63] Tuttle K. R., Bakris G. L., Toto R. D., McGill J. B., Hu K., Anderson P. W. (2005). The effect of ruboxistaurin on nephropathy in type 2 diabetes. *Diabetes Care*.

[64] Satchell S. C., Tooke J. E. (2008). What is the mechanism of microalbuminuria in diabetes: a role for the glomerular endothelium?. *Diabetologia*.

[65] Castellani P., Balza E., Rubartelli A. (2014). Inflammation, DAMPs, tumor development, and progression: a vicious circle orchestrated by redox signaling. *Antioxidants & Redox Signaling*.

[66] Mittal M., Siddiqui M. R., Tran K., Reddy S. P., Malik A. B. (2014). Reactive oxygen species in inflammation and tissue injury. *Antioxidants & Redox Signaling*.

[67] Biswas S. K. (2016). Does the interdependence between oxidative stress and inflammation explain the antioxidant paradox?. *Oxidative Medicine and Cellular Longevity*.

[68] Vaziri N. D., Rodríguez-Iturbe B. (2006). Mechanisms of disease: oxidative stress and inflammation in the pathogenesis of hypertension. *Nature Clinical Practice Nephrology*.

[69] Saraheimo M., Teppo A. M., Forsblom C., Fagerudd J., Groop P. H. (2003). Diabetic nephropathy is associated with low-grade inflammation in type 1 diabetic patients. *Diabetologia*.

[70] Moriwaki Y., Yamamoto T., Shibutani Y. (2003). Elevated levels of interleukin-18 and tumor necrosis factor-*α* in serum of patients with type 2 diabetes mellitus: Relationship with diabetic nephropathy. *Metabolism*.

[71] Dalla Vestra M., Mussap M., Gallina P. (2005). Acute-phase markers of inflammation and glomerular structure in patients with type 2 diabetes. *Journal of the American Society of Nephrology*.

[72] Dai S. M., Matsuno H., Nakamura H., Nishioka K., Yudoh K. (2004). Interleukin-18 enhances monocyte tumor necrosis factor alpha and interleukin-1beta production induced by direct contact with T lymphocytes: implications in rheumatoid arthritis. *Arthritis & Rheumatism*.

[73] Nakamura A., Shikata K., Hiramatsu M. (2005). Serum interleukin-18 levels are associated with nephropathy and atherosclerosis in Japanese patients with type 2 diabetes. *Diabetes Care*.

[74] Nakamura T., Fukui M., Ebihara I. (1993). mRNA expression of growth factors in glomeruli from diabetic rats. *Diabetes*.

[75] Luo S. F., Fang R. Y., Hsieh H. L. (2010). Involvement of MAPKs and NF-kappaB in tumor necrosis factor alpha-induced vascular cell adhesion molecule 1 expression in human rheumatoid arthritis synovial fibroblasts. *Arthritis & Rheumatism*.

[76] Sayed A. A., Khalifa M., Abd el-Latif F. F. (2012). Fenugreek attenuation of diabetic nephropathy in alloxan-diabetic rats: attenuation of diabetic nephropathy in rats. *Journal of Physiology and Biochemistry*.

[77] Xu G., Luo K., Liu H., Huang T., Fang X., Tu W. (2015). The progress of inflammation and oxidative stress in patients with chronic kidney disease. *Renal Failure*.

[78] Tucker P. S., Scanlan A. T., Dalbo V. J. (2015). Chronic kidney disease influences multiple systems: describing the relationship between oxidative stress, inflammation, kidney damage, and concomitant disease. *Oxidative Medicine and Cellular Longevity*.

[79] Yamagishi S., Matsui T. (2010). Advanced glycation end products, oxidative stress and diabetic nephropathy. *Oxidative Medicine and Cellular Longevity*.

[80] Bohlender J. M., Franke S., Stein G., Wolf G. (2005). Advanced glycation end products and the kidney. *American Journal of Physiology-Renal Physiology*.

[81] Kafle D., Signh N., Singh S. K., Singh N., Islam N. (2012). Relationship between hyperglycaemia, inflammation and oxidative stress in type2 diabetic nephropathy subjects. *International Journal of Pharmaceutical & Biological Archive*.

[82] Gnudi L. (2012). Cellular and molecular mechanisms of diabetic glomerulopathy. *Nephrology Dialysis Transplantation*.

[83] Mogensen C. E., Christensen C. K., Vittinghus E. (1983). The stages in diabetic renal disease. With emphasis on the stage of incipient diabetic nephropathy. *Diabetes*.

[84] Stephenson J. M., Fuller J. H. (1994). Microalbuminuria is not rare before 5 years of IDDM: EURODIAB IDDM Complications Study Group and the WHO Multinational Study of Vascular Disease in Diabetes Study Group. *Journal of Diabetes and its Complications*.

[85] Adler A. I., Stevens R. J., Manley S. E. (2003). Development and progression of nephropathy in type 2 diabetes: the United Kingdom Prospective Diabetes Study (UKPDS 64). *Kidney International*.

[86] Gross J. L., de Azevedo M. J., Silveiro S. P., Canani L. H., Caramori M. L., Zelmanovitz T. (2005). Diabetic nephropathy: diagnosis, prevention, and treatment. *Diabetes Care*.

[87] Selby N. M., Taal M. W. (2020). An updated overview of diabetic nephropathy: diagnosis, prognosis, treatment goals and latest guidelines. *Diabetes, Obesity and Metabolism*.

[88] American Diabetes Association (2019). 11. Microvascular complications and foot care: standards of medical care in diabetes—2019. *Diabetes Care*.

[89] Bermejo S., Pascual J., Soler M. J. (2017). The large spectrum of renal disease in diabetic patients. *Clinical Kidney Journal*.

[90] Satirapoj B. (2010). Review on pathophysiology and treatment of diabetic kidney disease. *Journal of the Medical Association of Thailand*.

[91] Koye D. N., Shaw J. E., Reid C. M., Atkins R. C., Reutens A. T., Magliano D. J. (2017). Incidence of chronic kidney disease among people with diabetes: a systematic review of observational studies. *Diabetic Medicine*.

[92] Rossing P., Hougaard P., Parving H. H. (2005). Progression of microalbuminuria in type 1 diabetes: ten-year prospective observational study. *Kidney International*.

[93] Robles N. R., Villa J., Felix F. J., Fernandez-Berges D., Lozano L. (2017). Non-proteinuric diabetic nephropathy is the main cause of chronic kidney disease: results of a general population survey in Spain. *Diabetes & Metabolic Syndrome: Clinical Research & Reviews*.

[94] Afkarian M., Zelnick L. R., Hall Y. N. (2016). Clinical manifestations of kidney disease among US adults with diabetes, 1988-2014. *JAMA*.

[95] Kume S., Araki S. I., Ugi S. (2019). Secular changes in clinical manifestations of kidney disease among Japanese adults with type 2 diabetes from 1996 to 2014. *Journal of Diabetes Investigation*.

[96] Pugliese G., Penno P., Natali A. (2020). Diabetic kidney disease: new clinical and therapeutic issues. Joint position statement of the Italian Diabetes Society and the Italian Society of Nephrology on “The natural history of diabetic kidney disease and treatment of hyperglycemia in patients with type 2 diabetes and impaired renal function”. *Journal of Nephrology*.

[97] de Boer I. H., Steffes M. W. (2007). Glomerular filtration rate and albuminuria: twin manifestations of nephropathy in diabetes. *Journal of the American Society of Nephrology*.

[98] Shimizu M., Furuichi K., Yokoyama H. (2014). Kidney lesions in diabetic patients with normoalbuminuric renal insufficiency. *Clinical and Experimental Nephrology*.

[99] Ekinci E. I., Jerums G., Skene A. (2013). Renal structure in normoalbuminuric and albuminuric patients with type 2 diabetes and impaired renal function. *Diabetes Care*.

[100] Yamanouchi M., Furuichi K., Hoshino J. (2019). Nonproteinuric versus proteinuric phenotypes in diabetic kidney disease: a propensity score-matched analysis of a nationwide, biopsy-based cohort study. *Diabetes Care*.

[101] Zoccali C., Mallamaci F. (2019). Nonproteinuric progressive diabetic kidney disease. *Current Opinion in Nephrology and Hypertension*.

[102] Chawla V., Roshan B. (2014). Non-proteinuric diabetic nephropathy. *Current Diabetes Reports*.

[103] MacIsaac R. J., Tsalamandris C., Panagiotopoulos S., Smith T. J., McNeil K. J., Jerums G. (2004). Nonalbuminuric renal insufficiency in type 2 diabetes. *Diabetes Care*.

[104] Silva R., Meng C., Coentrão L. (2017). Diabetic nephropathy and its two phenotypes: the proteinuric and non-proteinuric. *Portuguese Journal of Nephrology & Hypertension*.

[105] Thakar C. V., Christianson A., Himmelfarb J., Leonard A. C. (2011). Acute kidney injury episodes and chronic kidney disease risk in diabetes mellitus. *Clinical Journal of the American Society of Nephrology*.

[106] Sykes L., Asar O., Ritchie J. (2019). The influence of multiple episodes of acute kidney injury on survival and progression to end stage kidney disease in patients with chronic kidney disease. *PLoS One*.

[107] Sánchez-Lozada L. G., Lanaspa M. A., Cristóbal-García M. (2013). Uric acid-induced endothelial dysfunction is associated with mitochondrial alterations and decreased intracellular ATP concentrations. *Nephron Experimental Nephrology*.

[108] Rabadi M. M., Kuo M. C., Ghaly T. (2012). Interaction between uric acid and HMGB1 translocation and release from endothelial cells. *American Journal of Physiology-Renal Physiology*.

[109] Kang D. H., Park S. K., Lee I. K., Johnson R. J. (2005). Uric acid-induced C-reactive protein expression: implication on cell proliferation and nitric oxide production of human vascular cells. *Journal of the American Society of Nephrology*.

[110] Corry D. B., Eslami P., Yamamoto K., Nyby M. D., Makino H., Tuck M. L. (2008). Uric acid stimulates vascular smooth muscle cell proliferation and oxidative stress via the vascular renin-angiotensin system. *Journal of Hypertension*.

[111] Zhou Y., Fang L., Jiang L. (2012). Uric acid induces renal inflammation via activating tubular NF-*κ*B signaling pathway. *PLoS One*.

[112] Ryu E. S., Kim M. J., Shin H. S. (2013). Uric acid-induced phenotypic transition of renal tubular cells as a novel mechanism of chronic kidney disease. *American Journal of Physiology-Renal Physiology*.

[113] Niewczas M. A., Ficociello L. H., Johnson A. C. (2009). Serum concentrations of markers of TNFalpha and Fas-mediated pathways and renal function in nonproteinuric patients with type 1 diabetes. *Clinical Journal of the American Society of Nephrology*.

[114] Akcay A., Nguyen Q., Edelstein C. L. (2009). Mediators of inflammation in acute kidney injury. *Mediators of Inflammation*.

[115] Vielhauer V., Mayadas T. N. (2007). Functions of TNF and its receptors in renal disease: distinct roles in inflammatory tissue injury and immune regulation. *Seminars in Nephrology*.

[116] Ernandez T., Mayadas T. N. (2009). Immunoregulatory role of TN alpha in inflammatory kidney diseases. *Kidney International*.

[117] Esteghamati A., Arefzadeh A., Zandieh A., Salehi Sadaghiani M., Noshad S., Nakhjavani M. (2013). Comparison of osteoprotegerin and vascular endothelial growth factor in normoalbuminuric Type 1 diabetic and control subjects. *Journal of Endocrinological Investigation*.

[118] Buyadaa O., Magliano D. J., Salim A., Koye D. N., Shaw J. E. (2020). Risk of rapid kidney function decline, all-cause mortality, and major cardiovascular events in nonalbuminuric chronic kidney disease in type 2 diabetes. *Diabetes Care*.

[119] Fiorini F., Barozzi L. (2007). The role of ultrasonography in the study of medical nephropathy. *Journal of Ultrasound*.

[120] Abd el Dayem S., el Bohy AE, el Shehaby A. (2016). Value of the intrarenal arterial resistivity indices and different renal biomarkers for early identification of diabetic nephropathy in type 1 diabetic patients. *Journal of Pediatric Endocrinology and Metabolism*.

[121] Spatola L., Andrulli S. (2016). Doppler ultrasound in kidney diseases: a key parameter in clinical long-term follow-up. *Journal of Ultrasound*.

[122] Mancini M., Masulli M., Liuzzi R. (2013). Renal duplex sonographic evaluation of type 2 diabetic patients. *Journal of Ultrasound in Medicine*.

[123] Ruggenenti P., Fassi A., Ilieva A. P. (2005). Preventing microalbuminuria in type 2 diabetes. *ACC Current Journal Review*.

[124] Agarwal N., Sengar N. S., Jain P. K., Khare R. (2011). Nephropathy in newly diagnosed type 2 diabetics with special stress on the role of hypertension. *The Journal of the Association of Physicians of India*.

[125] Shestakova M. V., Koshel L. V., Vagodin V. A., Dedov I. (2006). Risk factors of diabetic nephropathy progression in patients with a long history of diabetic melitus as shown by a retrospective analysis. *Terapevticheskii arkhiv*.

[126] Lim A. K. H. (2014). Diabetic nephropathy—complications and treatment. *International Journal of Nephrology and Renovascular Disease*.

[127] Rohilla A., Tiwari S. K., Rohilla S., Kushnoor A. (2011). Diabetic nephropathy: pathogenesis, prevention and treatment. *European Journal of Experimental Biology*.

[128] Dronavalli S., Duka I., Bakris G. L. (2008). The pathogenesis of diabetic nephropathy. *Nature Clinical Practice Endocrinology & Metabolism*.

[129] Alicic R. Z., Rooney M. T., Tuttle K. R. (2017). Diabetic kidney disease: challenges, progress, and possibilities. *Clinical Journal of the American Society of Nephrology*.

[130] Doshi S. M., Friedman A. N. (2017). Diagnosis and management of type 2 diabetic kidney disease. *Clinical Journal of the American Society of Nephrology*.

[131] Nazar C. M. (2014). Diabetic nephropathy; principles of diagnosis and treatment of diabetic kidney disease. *Journal of Nephropharmacology*.

[132] de Zeeuw D., Remuzzi G., Parving H. H. (2004). Albuminuria, a therapeutic target for cardiovascular protection in type 2 diabetic patients with nephropathy. *Circulation*.

[133] Quiroga B., Arroyo D., de Arriba G. (2015). Present and future in the treatment of diabetic kidney disease. *Journal of Diabetes Research*.

[134] Eknoyan G. (2007). Obesity, diabetes, and chronic kidney disease. *Current Diabetes Reports*.

[135] Briffa J. F., McAinch A. J., Poronnik P., Hryciw D. H. (2013). Adipokines as a link between obesity and chronic kidney disease. *American Journal of Physiology-Renal Physiology*.

[136] Stratton I. M., Adler A. I., Neil H. A. (2000). Association of glycaemia with macrovascular and microvascular complications of type 2 diabetes (UKPDS 35): prospective observational study. *BMJ*.

[137] for the ADVANCE Collaborative Group, Zoungas S., Chalmers J. (2012). Association of HbA1c levels with vascular complications and death in patients with type 2 diabetes: evidence of glycaemic thresholds. *Diabetologia.*.

[138] American Diabetes Association (2016). 5. Glycemic targets. *Diabetes Care*.

[139] National Kidney Foundation (2012). KDOQI clinical practice guideline for diabetes and CKD: 2012 update. *American Journal of Kidney Diseases*.

[140] Bailie G. R., Eisele G., Liu L. (2005). Patterns of medication use in the RRI-CKD study: focus on medications with cardiovascular effects. *Nephrology Dialysis Transplantation*.

[141] Balant L., Zahnd G., Gorgia A., Schwarz R., Fabre J. (1973). Pharmacokinetics of glipizide in man: influence of renal insufficiency. *Diabetologia*.

[142] Palmer K. J., Brogden R. N. (1993). Gliclazide. An update of its pharmacological properties and therapeutic efficacy in non-insulin-dependent diabetes mellitus. *Drugs*.

[143] Arnouts P., Bolignano D., Nistor I. (2014). Glucose-lowering drugs in patients with chronic kidney disease: a narrative review on pharmacokinetic properties. *Nephrology Dialysis Transplantation*.

[144] Neumiller J. J., Alicic R. Z., Tuttle K. R. (2017). Therapeutic considerations for antihyperglycemic agents in diabetic kidney disease. *Journal of the American Society of Nephrology*.

[145] Marbury T. C., Ruckle J. L., Hatorp V. (2000). Pharmacokinetics of repaglinide in subjects with renal impairment. *Clinical Pharmacology & Therapeutics*.

[146] Hahr A. J., Molitch M. E. (2015). Management of diabetes mellitus in patients with chronic kidney disease. *Clinical Diabetes and Endocrinology*.

[147] Graham G. G., Punt J., Arora M. (2011). Clinical pharmacokinetics of metformin. *Clinical Pharmacokinetics*.

[148] Drucker D. J., Nauck M. A. (2006). The incretin system: glucagon-like peptide-1 receptor agonists and dipeptidyl peptidase-4 inhibitors in type 2 diabetes. *Lancet*.

[149] Panchapakesan U., Pollock C. (2015). The role of dipeptidyl peptidase-4 inhibitors in diabetic kidney disease. *Frontiers in Immunology*.

[150] Zhong J., Rao X., Rajagopalan S. (2013). An emerging role of dipeptidyl peptidase 4 (DPP4) beyond glucose control: potential implications in cardiovascular disease. *Atherosclerosis*.

[151] Wolf G., Ziyadeh F. N. (2007). Cellular and Molecular Mechanisms of Proteinuria in Diabetic Nephropathy. *Nephron Physiology*.

[152] Tiruppathi C., Miyamoto Y., Ganapathy V., Roesel R. A., Whitford G. M., Leibach F. H. (1990). Hydrolysis and transport of proline-containing peptides in renal brush-border membrane vesicles from dipeptidyl peptidase IV-positive and dipeptidyl peptidase IV-negative rat strains. *Journal of Biological Chemistry*.

[153] Mentlein R. (1999). Dipeptidyl-peptidase IV (CD26)—role in the inactivation of regulatory peptides. *Regulatory Peptides*.

[154] Kim M. K. (2017). Treatment of diabetic kidney disease: current and future targets. *The Korean Journal of Internal Medicine*.

[155] Wanner C., Inzucchi S. E., Lachin J. M. (2016). Empagliflozin and progression of kidney disease in type 2 diabetes. *New England Journal of Medicine*.

[156] Katz P. M., Leiter L. A. (2015). The role of the kidney and SGLT2 inhibitors in type 2 diabetes. *Canadian Journal of Diabetes*.

[157] Vallon V., Gerasimova M., Rose M. A. (2014). SGLT2 inhibitor empagliflozin reduces renal growth and albuminuria in proportion to hyperglycemia and prevents glomerular hyperfiltration in diabetic Akita mice. *American Journal of Physiology-Renal Physiology*.

[158] De Nicola L., Gabbai F. B., Liberti M. E., Sagliocca A., Conte G., Minutolo R. (2014). Sodium/glucose cotransporter 2 inhibitors and prevention of diabetic nephropathy: targeting the renal tubule in diabetes. *American Journal of Kidney Diseases*.

[159] Froett M. A., Liegl S., Jabbarpour Y. (2012). Diabetic nephropathy—the family physician’s role. *American Family Physician*.

[160] American Diabetes Association (2016). 9. Microvascular complications and foot care. *Diabetes Care*.

[161] Taler S. J., Agarwal R., Bakris G. L. (2013). KDOQI US Commentary on the 2012 KDIGO Clinical Practice Guideline for Management of Blood Pressure in CKD. *American Journal of Kidney Diseases*.

[162] Becker G. J., Wheeler D. C., De Zeeuw D. (2012). Kidney disease: Improving global outcomes (KDIGO) blood pressure work group. KDIGO clinical practice guideline for the management of blood pressure in chronic kidney disease. *Kidney International Supplements*.

[163] Umanath K., Lewis J. B. (2018). Update on diabetic nephropathy: CoreCurriculum 2018. *American Journal of Kidney Diseases*.

[164] Zac-Varghese S., Winocour P. (2018). Managing diabetic kidney disease. *British Medical Bulletin*.

[165] Brem A. S., Morris D. J., Gong R. (2011). Aldosterone-induced fibrosis in the kidney: questions and controversies. *American Journal of Kidney Diseases*.

[166] Saklayen M. G., Gyebi L. K., Tasosa J., Yap J. (2008). Effects of additive therapy with spironolactone on proteinuria in diabetic patients already on ACE inhibitor or ARB therapy: results of a randomized, placebo-controlled, double-blind, crossover trial. *Journal of Investigative Medicine*.

[167] Davidson M. B., Wong A., Hamrahian A. H., Stevens M., Siraj E. S. (2008). Effect of spironolactone therapy on albuminuria in patients with type 2 diabetes treated with angiotensin-converting enzyme inhibitors. *Endocrine Practice*.

[168] Mehdi U. F., Adams-Huet B., Raskin P., Vega G. L., Toto R. D. (2009). Addition of angiotensin receptor blockade or mineralocorticoid antagonism to maximal angiotensin-converting enzyme inhibition in diabetic nephropathy. *Journal of the American Society of Nephrology*.

[169] Gagliardini E., Zoja C., Benigni A. (2015). Et and diabetic nephropathy: preclinical and clinical studies. *Seminars in Nephrology*.

[170] Mann J. F., Green D., Jamerson K. (2010). Avosentan for overt diabetic nephropathy. *Journal of the American Society of Nephrology*.

[171] Dusso A. S., Brown A. J., Slatopolsky E. (2005). Vitamin D. *American Journal of Physiology-Renal Physiology*.

[172] Li Y. C., Qiao G., Uskokovic M., Xiang W., Zheng W., Kong J. (2004). Vitamin D: a negative endocrine regulator of the renin-angiotensin system and blood pressure. *The Journal of Steroid Biochemistry and Molecular Biology*.

[173] Pérez-Gómez M. V., Ortiz-Arduán A., Lorenzo-Sellares V. (2013). Vitamin D and proteinuria: a critical review of molecular bases and clinical experience. *Nefrologia*.

[174] Chokhandre M. K., Mahmoud M. I., Hakami T., Jafer M., Inamdar A. S. (2015). Vitamin D & its analogues in type 2 diabetic nephropathy: a systematic review. *Journal of Diabetes & Metabolic Disorders*.

[175] Fernández-Juárez G., Luño J., Barrio V. (2013). 25(OH) vitamin D levels and renal disease progression in patients with type 2 diabetic nephropathy and blockade of the renin-angiotensin system. *Clinical Journal of the American Society of Nephrology*.

[176] de Borst M. H., Hajhosseiny R., Tamez H., Wenger J., Thadhani R., Goldsmith D. J. (2013). Active vitamin D treatment for reduction of residual proteinuria: a systematic review. *Journal of the American Society of Nephrology*.

[177] Wang Y., Deb D. K., Zhang Z. (2012). Vitamin D receptor signaling in podocytes protects against diabetic nephropathy. *Journal of the American Society of Nephrology*.

[178] Lei M., Liu Z., Guo J. (2020). The emerging role of vitamin D and vitamin D receptor in diabetic nephropathy. *BioMed Research International*.

[179] Larsson T., Nisbeth U., Ljunggren O., Juppner H., Jonsson K. B. (2003). Circulating concentration of FGF-23 increases as renal function declines in patients with chronic kidney disease, but does not change in response to variation in phosphate intake in healthy volunteers. *Kidney International*.

[180] McCormick B. B., Sydor A., Akbari A., Fergusson D., Doucette S., Knoll G. (2008). The effect of pentoxifylline on proteinuria in diabetic kidney disease: a meta-analysis. *American Journal of Kidney Diseases*.

[181] Ghorbani A., Omidvar B., Beladi-Mousavi S. S., Lak E., Vaziri S. (2012). The effect of pentoxifylline on reduction of proteinuria among patients with type 2 diabetes under blockade of angiotensin system: a double blind and randomized clinical trial. *Nefrologia*.

[182] Navarro-González J. F., Mora-Fernández C., Muros de Fuentes M. (2015). Effect of pentoxifylline on renal function and urinary albumin excretion in patients with diabetic kidney disease: the PREDIAN trial. *Journal of the American Society of Nephrology*.

[183] Moreno J. A., Moreno S., Rubio-Navarro A. (2012). Targeting chemokines in proteinuria-induced renal disease. *Expert Opinion on Therapeutic Targets*.

[184] de Zeeuw D., Bekker P., Henkel E. (2015). The effect of CCR2 inhibitor CCX140-B on residual albuminuria in patients with type 2 diabetes and nephropathy: a randomised trial. *The Lancet Diabetes & Endocrinology*.

[185] Daenen K., Andries A., Mekahli D., Van Schepdael A., Jouret F., Bammens B. (2019). Oxidative stress in chronic kidney disease. *Pediatric Nephrology*.

[186] Pizzino G., Irrera N., Cucinotta M. (2017). Oxidative stress: harms and benefits for human health. *Oxidative Medicine and Cellular Longevity*.

[187] Saha S. K., Lee S. B., Won J. (2017). Correlation between oxidative stress, nutrition, and cancer initiation. *International Journal of Molecular Sciences*.

[188] Galle J., Schwedhelm E., Pinnetti S., Böger R. H., Wanner C., VIVALDI investigators (2008). Antiproteinuric effects of angiotensin receptor blockers: telmisartan versus valsartan in hypertensive patients with type 2 diabetes mellitus and overt nephropathy. *Nephrology Dialysis Transplantation*.

[189] Sugiyama H., Kobayashi M., Wang D. H. (2005). Telmisartan inhibits both oxidative stress and renal fibrosis after unilateral ureteral obstruction in acatalasemic mice. *Nephrology Dialysis Transplantation*.

[190] Takaya T., Kawashima S., Shinohara M. (2006). Angiotensin II type 1 receptor blocker telmisartan suppresses superoxide production and reduces atherosclerotic lesion formation in apolipoprotein E-deficient mice. *Atherosclerosis*.

[191] Kitada M., Koya D. (2013). Renal protective effects of resveratrol. *Oxidative Medicine and Cellular Longevity*.

[192] Qiao Y., Gao K., Wang Y., Wang X., Cui B. (2017). Resveratrol ameliorates diabetic nephropathy in rats through negative regulation of the p38 MAPK/TGF-*β*1 pathway. *Experimental and Therapeutic Medicine*.

[193] Kitada M., Kume S., Imaizumi N., Koya D. (2011). Resveratrol improves oxidative stress and protects against diabetic nephropathy through normalization of Mn-SOD dysfunction in AMPK/SIRT1-independent pathway. *Diabetes*.

[194] Zheng H., Whitman S. A., Wu W. (2011). Therapeutic potential of Nrf2 activators in streptozotocin-induced diabetic nephropathy. *Diabetes*.

[195] Ruiz S., Pergola P. E., Zager R. A., Vaziri N. D. (2013). Targeting the transcription factor Nrf2 to ameliorate oxidative stress and inflammation in chronic kidney disease. *Kidney International*.

[196] Pergola P. E., Raskin P., Toto R. D. (2011). Bardoxolone methyl and kidney function in CKD with type 2 diabetes. *New England Journal of Medicine*.

[197] de Zeeuw D., Akizawa T., Audhya P. (2013). Bardoxolone methyl in type 2 diabetes and stage 4 chronic kidney disease. *New England Journal of Medicine*.

[198] Gold R., Kappos L., Arnold D. L. (2012). Placebo-controlled phase 3 study of oral BG-12 for relapsing multiple sclerosis. *New England Journal of Medicine*.

[199] Perez-Gomez M. V., Sanchez-Niño M. D., Sanz A. B. (2015). Horizon 2020 in diabetic kidney disease: the clinical trial pipeline for add-on therapies on top of renin angiotensin system blockade. *Journal of Clinical Medicine*.

